The article "Analysis of the Effect of Holistic Nursing in the Operating Room Based on PDCA and Evidence-Based Nursing in the Otorhinolaryngology Operating Room: Based on a Retrospective Case-Control Study" was retracted in 2023. Reasons: unreliable results or conclusions; lack of ethics approval or compliance; concerns about the data; concerns about the peer review.

# Analysis of the Effect of Holistic Nursing in the Operating Room Based on PDCA and Evidence-Based Nursing in the Otorhinolaryngology Operating Room: Based on a Retrospective Case-Control Study

**DOI:** 10.1155/2022/4514669

**Published:** 2022-05-21

**Authors:** Leina Bian, Jianhua Li, Wang Li, Xiaoyan Hu, Ming Dai

**Affiliations:** ^1^First People's Hospital Through the Operation Room, 222000 Lianyungang, China; ^2^First People's Hospital Conduit Room, 222000 Lianyungang, China

## Abstract

**Objective:**

Based on a retrospective case-control study, this study aims to explore the effect of holistic nursing in operating room based on PDCA (plan, do, check, and action) process and evidence-based nursing (EBN) in a ear, nose, and throat operating room.

**Methods:**

About 200 patients who underwent otorhinolaryngology surgery in our hospital from January 2019 to September 2021 were enrolled. According to the difference of nursing mode, patients were assigned into a control group and study group; holistic nursing in operating room was included in control group, and holistic nursing in the operating room based on PDCA and EBN was included in study group. Nursing satisfaction, hypothermia, chills, restlessness, related indexes of operating room, nursing quality scores of operating room, and individual quality control scores were compared.

**Results:**

First of all, we compared the nursing satisfaction, the study group was very satisfied in 69 cases, satisfactory in 30 cases, general in 1 case, the satisfaction rate was 100.00%, while in the control group, 46 cases were very satisfied, 34 cases were satisfied, 13 cases were general, and 7 cases were dissatisfied, the satisfaction rate was 93.00%. The nursing satisfaction of the study group was higher compared to the control group (*P* < 0.05). Second, we compared the incidence of hypothermia, chills and restlessness. The incidence of hypothermia, chills, and restlessness in the study group was lower compared to the control group (*P* < 0.05). The time of tracheal tube extubation, PACU stay time, postoperative hospitalization time, hospitalization cost, and operation time in the study group was significantly lower compared to the control group (*P* < 0.05). In terms of the scores of nursing quality in the operating room, the instruments and equipment management, equipment preparation, nurses' cooperation skills, disinfection and isolation quality, and total score in the study group were higher compared to the control group (*P* < 0.05). Finally, we compared the scores of individual quality control examination. The scores of ward management, rescue, therapeutic articles, drug management, first-level nursing, nursing documents, and head nurse management in the study group were higher compared to the control group (*P* < 0.05).

**Conclusion:**

Incorporating the concepts of PDCA and EBN into the overall care of the operating theatre is effective for patients in the ENT operating theatre. Our results show that this care can be effective in improving patients' surgical indicators, reducing the incidence of postoperative infections, shortening postoperative resuscitation and length of stay, reducing hospital costs, and promoting surgical patient satisfaction. While further multicenter studies are necessary, this series of nursing interventions remains worthy of replication in the clinical setting.

## 1. Introduction

Ear, nose, and throat diseases can be summarized as trauma, congenital abnormal mutation, infection, tumor phenomenon, and foreign body entry, etc. The head and neck region of ear, nose, and throat is the necessary passage of respiratory tract or digestive tract, multiple foreign bodies, and infection [1]. It is also a frequent site of benign or malignant tumors. In addition, congenital ear malformations caused by genetic or environmental factors are the most common [2]. The common clinical symptoms include otitis media, tympanic membrane perforation, and tympanic membrane repair in ear diseases, nasal diseases including inflammation of nose and paranasal sinuses and nasal polyps, and throat diseases including inflammation of pharynx and larynx, adenoid hypertrophy, tonsillitis, and polyps in vocal cords [3]. Clinically, because the nose and ear are connected with each other through the eustachian tube, when inflammation occurs in the nose, it will cause edema of the nasal mucosa, in which case the eustachian tube will be blocked. Because the external gas cannot enter the tympanum normally and in time, it may cause the blood vessels of the middle ear mucosa to dilate and produce congestion, leading to the occurrence of otitis media [4]. In medicine, the parietal wall of the middle ear is called the tympanic cover. After dissection, it can be observed that there is only a thin bone wall between the tympanum and the brain, and it is also very close to the cerebellum [3, 4]. Once the disease of the middle ear occurs, such as severe inflammation, the bone will be infected or damaged. At this time, the infected microorganisms may enter the human skull, and in serious cases, bring meningitis, which may cause very serious consequences. Therefore, any infection in the ear, nose, and throat may cause pathological changes in other parts. If you suffer from related diseases, you must seek medical treatment in time to avoid causing other emergencies and increase the burden on patients [5]. As we known, otorhinolaryngological diseases are common in clinic, including otitis media, tympanic membrane perforation and tympanic membrane repair, nasal diseases including rhinitis, sinusitis, and nasal polyps, etc. On the other hand, pharynx and throat diseases include pharyngitis, adenoid hypertrophy, tonsillitis, and vocal cord polyps. These symptoms seriously affect the life quality of patients and healthy people. Clinical treatment of otorhinolaryngological diseases is mostly with the help of surgery because the hospital environment is complex, there are many pathogens; in addition, clinical otorhinolaryngological diseases have particularity. Postoperative infection is not only a high incidence of postoperative complications in otorhinolaryngology but also a key index to reflect nosocomial infection [6].

The quality of nursing in operating room is the quality of nursing work with medical treatment as the core, which reflects the comprehensive effect of all kinds of activities in the hospital and the level to meet the requirements [7]. The nursing quality of the operating room is the main component of the hospital quality. In principle, the nursing quality of the operating room is mainly reflected in the medical quality. The quality of nursing in the operating room is directly related to the health and life of patients, which is not only the key to the survival and development of the hospital but also the focus of social attention [8]. Nursing in operating room runs through the whole process of surgical treatment, which directly affects the effect of operation and is closely related to the prognosis of patients. Holistic nursing in operating room has received clinical attention, but there are some problems in the process of implementation: the concept of nursing is backward and the scope of knowledge is narrow [9]. Subjectively, most nurses' understanding of nursing in the operating room still stays in the traditional passive operation, but they do not know much about the individual needs of patients. Unable to actively and effectively communicate with patients and provide complete health education, holistic nursing in the operating room is difficult to implement. Many studies pointed out that the scope of operating room visits and health education is narrow, lack of postoperative rehabilitation education, lack of professionalism, lack of special disease interviews and operating room specialty characteristics, lack of evidence-based basis, and do not understand the cutting-edge technologies and concepts of surgery [8, 9]. The phenomenon that the visiting object is single. EBN is a new clinical nursing concept, model, or nursing methodology with the rapid development of evidence-based medicine (EBM) in the past 10 years. However, some research institutions in Canada, Britain, and Australia were the first to use EBM in nursing work. Its core is to suggest that nursing staff should not deal with problems solely on the basis of clinical experience or outdated or imperfect theoretical knowledge in practice, but should follow scientific principles and basis. In recent years, some mature application of PDCA (plan, do, check, and action) process is represented by nursing quality management: some scholars apply PDCA cycle to hospital nursing staff education, which greatly improves the satisfaction of nursing staff. Some scholars also use the PDCA circulation method to improve the blood glucose detection method of inpatients and improve the level of nursing quality [9]. Some studies have pointed out that there is a high incidence of perioperative hypothermia in patients undergoing otorhinolaryngology. The data reported in a cross-sectional survey in some areas of the country in 2017 are 44.5% [10]. Intraoperative pressure sore nursing, perioperative prevention, and treatment of venous thromboembolism are also hot issues in the development of specialization in operating rooms in recent years. PDCA and EBN concepts are integrated into holistic nursing and applied to surgical patients. It can not only promote the overall nursing care of patients in the operating room but also enhance the speed and quality of perioperative rehabilitation to improve the prognosis.

## 2. Patients and Methods

### 2.1. General Information

About 200 patients who underwent otorhinolaryngology surgery in our hospital from January 2019 to September 2021 were enrolled. According to the difference of nursing mode, patients were assigned into control group and study group. Holistic nursing in operating room was included in control group, and holistic nursing in operating room based on PDCA and EBN was included in study group. In the control group, the age was from 15 to 78 years old, with an average age of 45.43 ± 3.34 years, including 56 males and 44 females, while in the study group, the age was from 16 to 79 years old, with an average age of 45.67 ± 3.33 years, including 53 males and 47 females. No statistical significance was exhibited in the general data.

Inclusion criteria were as follows: (1) those who had the indication of otorhinolaryngological surgery and (2) those who had no cognitive, language and intellectual impairment, and have basic reading and writing ability.

Exclusion criteria were as follows: (1) those with severe heart, liver, renal insufficiency, malignant tumors, and other diseases and (2) those who refused to participate.

### 2.2. Treatment Methods

The control group received holistic nursing care in the operating room: (1) the day before operation, the itinerant nurses of the specialist group and the anesthesiologist visited the ward together. On the basis of routine visits, the specialist knowledge was integrated, and the flow communication mode (CICARE) was adopted, including C (Connect) contact, I (Introduce) introduction, C (Communicate) communication, A (Ask) inquiry, R (Respond) answer, and E (Exit) leave these six processes. The contents of the interview are as follows:

1. Politely address patients and their families, encourage patients' families to participate in the visit process, explain the differences and advantages between laparoscopic surgery and traditional surgery, introduce the surgical team of this study, and share successful cases. Relieve patients' fear and anxiety;
2. Explain the operation procedure and related operation significance, so that patients and their families can have a better understanding of the information of the operation process;
3. Inform patients that they can eat normally 6 hours before operation, and take 400 ml of carbohydrates 2 hours before operation (except for patients with gastrointestinal motility disturbance). There is no need for intestinal preparation, and chewing gum can be chewed after operation;
4. Accurately evaluate the patients, implement graded pain relief, encourage patients to correctly express pain and actively cooperate with postoperative functional training, such as breathing exercise, effective cough, ankle pump exercise, straight leg raising exercise;
5. Perioperative hypothermia (<36°C) risk assessment was carried out according to the patients' age, BMI index, preoperative basic body temperature and operative factors, so as to facilitate the active heat preservation of the patients at each stage during the operation. Meanwhile, the Caprini score scale was used to assess the risk of venous thrombosis, and the corresponding nursing measures were drawn up according to the evaluation scores before operation;
6. Ask the patients what other information they want to know, encourage them to express their psychological needs, respect them, and thank them for their cooperation when they leave at the end of the visit.
7. Detail nursing: give more companionship, communication and distraction to nervous and anxious patients; inform patients during puncture and other operations, carry out painless operation as far as possible, and meanwhile pay attention to protect patients' privacy; wipe off wound disinfectant and blood stains after operation. Body temperature management: 30 minutes before the operation patient enters the operating room, adjust the room temperature to 22∼24°C, open the heating blanket in advance to pre-insulate the operation bed, heat up the intravenous infusion, keep the catheter for temperature measurement after anesthesia, and monitor the body temperature every 15 minutes. Avoid exposure to non-disinfection areas and keep warm with sheets, raise room temperature properly during skin disinfection, and use 39∼40°C abdominal lavage fluid during operation. (3) Routinely use warm air blanket to keep warm, regularly monitor body temperature and keep body temperature around 36.5°C. Closely observe the recovery of heart rate, blood pressure, blood oxygen saturation, consciousness, muscle strength, and respiration. Try to avoid the occurrence of moderate and severe pain, chills, restlessness, nausea, and vomiting. Use encouraging language to wake-up patients with spontaneous breathing, inform them that the operation has been completed successfully, and let them open their eyes. Take a good breath, the endotracheal tube will be removed quickly, and the patient will be in a suitable position for conscious observation.

Study group based on PDCA and EBN concept of operating room holistic nursing: operating room holistic nursing with the control group, based on PDCA and EBN concepts are as follows: (1) PDCA concept: PDCA circulation method as a universal work procedure, also known as Dai Minhuan. The letters P, D, C, and A represent four processes: P (plan) is the planning stage, through the analysis of the current situation to find out the existing problems, and put forward the corresponding solutions; D (do) is the implementation stage, the implementation of the P phase of the plan; C (check) is the inspection phase, tracking the implementation of the plan. A (action) is the processing stage, summing up the problems found by the inspection in stage C is the end of the first cycle and the beginning of the next cycle. It is necessary to make clear what problems have been solved and which problems need to be solved, will correctly form the standard work flow, and enter the next cycle that needs to be demonstrated. Through reciprocating cycles, continuous quality improvement is carried out to form a stepped ascending process. (2) The concept of EBN: (1) to find the problems in clinical practice and their specific structure; systematic review of the relevant literature to find external evidence based on the questions raised. The effectiveness of scientific evidence and promote careful review; (2) the obtained research evidence and clinical professional knowledge and experience, patient needs, combined with research to clinical evidence, according to clinical evidence to meet the needs of patient care plan; the realization effect of clinical evidence; (3) through self-evaluation, peer review and review, the implementation effect of clinical evidence is monitored. With the in-depth understanding of EBN of nursing and clinical nurses in our country, we begin to integrate EBN methods and nursing practice, promote the development of nursing science in our country and play a positive role, bring direct benefits to patients, reduce hospitalization costs, and put forward new requirements for EBN.

### 2.3. Observation Index

#### 2.3.1. Satisfaction

After consulting the literature and experts' discussion, we designed patients' follow-up satisfaction, a total of 10 items, and recorded patients' satisfaction with follow-up management mode, health education, medical and nursing service, and appointment registration process [11]. It is assigned into four dimensions: very satisfied, satisfied, general, and dissatisfied. Satisfaction rate = very satisfaction rate + satisfaction rate + general rate.

#### 2.3.2. Incidence of Hypothermia, Chills, and Restlessness

The incidences of hypothermia, chills and restlessness were recorded.

#### 2.3.3. Related Index of the Operating Room

The tracheal tube extubation time, PACU stay time, postoperative hospitalization time, hospitalization cost, and operation time were calculated.

#### 2.3.4. Incidence of Postoperative Infection

The incidences of respiratory tract infection, urinary tract infection, digestive tract infection, and other infections were calculated.

#### 2.3.5. Nursing Quality Score in the Operating Room

Nursing quality score of the operating room [12]: one day after the operation, the head nurse regularly scored the nursing quality of the whole operation process, including equipment management, equipment preparation, nurses' cooperation skills, disinfection and isolation quality, and the total score. The full score is 100, and the higher the score, the better the nursing quality in the operating room.

#### 2.3.6. Score of Individual Quality Control Examination in Clinical Departments

This paper uses the “Evaluation Standard of Nursing quality Control in Clinical Department,” which is being employed by the nursing department of this hospital in the assessment of nursing quality in clinical department, as the evaluation index. The evaluation standard is the standard of nursing quality management revised by the members of the joint nursing expert supervision group of the nursing department of the hospital with reference to “Evaluation Indexes of the third-level General Hospital of the Ministry of Health” [13] and (JCI Certification and quality Hospital Evaluation Indexes” [14]), combined with the actual situation of clinical nursing work. The standard divides the nursing quality management of clinical departments into five dimensions. Among them, the ward management mainly examines the clinical nurses' mastery of basic nursing; the quality management standards of rescue, and treatment materials/drugs mainly assess the management of necessary equipment and drugs in the ward; special first-level nursing management mainly evaluates whether nurses can provide timely, effective holistic nursing for critically ill patients; nursing document management mainly evaluates whether nurses can record the nursing process according to the standards. The higher the score, the better the effect of individual quality control examination in the clinical department.

### 2.4. Statistical Analysis

In the statistical processing, the data were analyzed by SPSS22.0 statistical software package. The counting data were presented by the number of cases (*n*) and the rate (%), the chi-square test was employed, the measurement data were presented by *t*-test, the continuous variables were presented by the method of mean ± standard deviation, and the data in accordance with normal distribution are presented by analysis of variance. The correlation between variables was tested by linear correlation test, and all statistical analysis indicated that there exhibited significant difference (*P* < 0.05), which was statistically significant.

## 3. Results

### 3.1. Nursing Satisfaction of Two Different Groups

First of all, we compared the nursing satisfaction. The study group was very satisfied in 69 cases, satisfactory in 30 cases, general in 1 case, and the satisfaction rate was 100.00%. The control group was very satisfied in 46 cases, satisfactory in 34 cases, general in 13 cases, and dissatisfied in 7 cases, the satisfaction rate was 93.00%. The nursing satisfaction in the study group was higher compared to the control group (*P* < 0.05). All the data results are indicated in Figure 1.

### 3.2. Incidence of Hypothermia, Chills, and Restlessness between Two Groups

Second, we compared the incidence of hypothermia, chills and restlessness. The incidence of hypothermia, chills, and restlessness in the study group was lower compared to the control group (*P* < 0.05). All the data results are indicated in Figure 2.

### 3.3. Related Indexes in the Operating Room between Two Groups

Third, we compared the relevant indexes of the operating room. The tracheal tube extubation time, PACU stay time, postoperative hospital stay, hospitalization expenses, and operation time in the study group were lower compared to the control group (*P* < 0.05). All the data results are indicated in Table 1.

### 3.4. Incidence of Postoperative Infection between Different Two Groups

Then, we compared the incidence of postoperative infection. The incidence of respiratory tract infection, urinary tract infection, digestive tract infection, and other infections in the study group was lower compared to the control group (*P* < 0.05). All the data results are indicated in Figure 3.

### 3.5. Comparison of Nursing Quality Score in the Operating Room

Next, we compared the nursing quality scores. The equipment management, equipment preparation, nurses' cooperation skills, disinfection and isolation quality, and total score of the study group were higher compared to the control group (*P* < 0.05). All the data results are indicated in Table 2.

### 3.6. Comparison of Individual Quality Control Examination Scores in Clinical Departments

Finally, we compared the scores of individual quality control examination. The scores of ward management, rescue, therapeutic articles, drug management, first-level nursing, nursing documents, and head nurse management in the study group were higher compared to the control group (*P* < 0.05). All the data results are indicated in Table 3.

## 4. Discussion

At present, with the continuous progress of social science and technology, medical devices, and technology have been continuously developed [13]. Otorhinolaryngological diseases are more frequent clinical diseases, and the quality of life of human beings is also tortured and affected by these diseases. Surgical treatment is often adopted in clinics [14]. Because of the complex hospital environment, many kinds of pathogens and the particularity of otorhinolaryngology diseases, postoperative infection is a postoperative complication with a high incidence in otorhinolaryngology. Once infection occurs, it will prolong the cure time of patients, increase the medical expenses of patients, and prolong the rehabilitation process, which will not only increase the economic burden of patients [15]. There are many factors affecting infection after otorhinolaryngology surgery, but there are few studies on the isolation and identification of pathogens causing infection, and mainly bacteria, and with the continuous increase of multiple drug-resistant bacteria, clinical control of pathogenic microorganisms causing infection is becoming more difficult, so timely and early detection and control of these pathogens will be of great help for clinicians to control patients' infection [16]. Regarding otorhinolaryngological surgery with other clinical diseases, it can be found that otorhinolaryngological surgery is easy to cause infectious complications. It will have a great impact on the rapid recovery of patients and the quality of life [16]. The factors related to postoperative infection in otorhinolaryngology surgery are complex and diverse, including nursing care of clinical doctors and nurses, use of antibiotics, aseptic operating environment, time of surgical treatment, and location of surgical treatment, etc. Among them, the operation time is the first important factor leading to infection after otorhinolaryngological surgery because the longer the time of surgical treatment, the longer the exposure time of surgical treatment. The chance of pathogens in the environment infecting patients will be greatly increased. The abuse and overuse of antibiotics have also increased the rate of nosocomial infection, especially in recent years, bacterial drug resistance has become more serious [17]. It has been reported that stress response factors can also bring about a decline in immune function, increase susceptibility to infection and reduce resistance [18].

Under the guidance of the modern nursing concept, holistic nursing in the operating room forms a planned and systematic specific nursing procedure, which provides the best nursing for surgical patients according to their physiological, psychological, social, cultural, and spiritual needs, including preoperative visit, intraoperative nursing, postoperative follow-up; however, a single operating room holistic nursing cannot meet the current otorhinolaryngological operating room nursing needs [19]. PDCA process is the abbreviation of plan, do, check and action in English. It was put forward by Dr. Deming, an American quality management expert, in the 1950s. It is the basic method of total quality management [20]. The PDCA process is assigned into four stages: planning stage, implementation stage, inspection stage, and treatment stage. These four stages are often carried out. In practical work, the specific operation is usually indicated as follows: first setting the work goal or raising the problem, then analyzing the problem, finding out the cause and then formulating measures, implementing measures in the process of implementation while checking the implementation effect while summing up the experience to transfer to the next cycle, is an effective management method of continuous improvement spiraling [21]. In the past decade, the clinical nursing practice in most countries in the world has undergone great changes. The concept based on evidence-based evidence has been accepted and accepted by many medical workers. EBN is an important branch of EBM. Its core is to develop traditional nursing based on experience and modern nursing based on science [22]. EBN is a nursing concept, which is influenced by the concept of EBM in the 1990s. This is a new concept of clinical nursing, which, like holistic nursing, has gradually penetrated into all fields of nursing work [23]. In the 1970s, Cochran, a British epidemiologist, believed that the practice of health care should be based on reasonable evidence, rather than on traditional subjective experience. In 1991, Canadian scholar Gates first put forward the term “EBM.” With the misunderstanding of the concept of EBN and the search of the literature on EBN in recent years, we can find that some nursing based on EBN is called “new theory” and “new nursing model.” And some EBN literature is called “new nursing discipline.” EBN was first put forward by Professor Alba Diconso of Ma Master University in Canada in 1991. Since then, nursing experts have been trying to enhance the system of EBN, popularizing and applying the concept of EBN [24]. When the concept of EBN has not been deeply rooted in the hearts of the people, their thought has gone through a long period of development. In order to make the concept of EBN accepted and recognized by a large number of nursing scholars, researchers made a lot of efforts at the initial stage when the concept of EBN was widely accepted, from abroad to home, EBN was in Canada in 1992, the United Kingdom in 1993, the United Kingdom in 1996 and Australia in 1997. Moreover, China, in March 1997 both spread and spread, and made historic breakthroughs [25]. In 1996, at the University of York in the United Kingdom, they launched and implemented the first “EBN” center, and they made phased progress and breakthrough in this field. However, they did not widely apply this concept of EBN to clinical practice. Then, our second evidence-based care center was established in Australia in 1997, and the establishment of this evidence-based care center has caused varying degrees of response and resonance all over the world [26, 27]. In March 1997, under the influence of advanced ideas, the Ministry of Health of China established the Cochrane Center of follow-up Medicine, which is located in West China Hospital of Sichuan University [28]. Therefore, on this basis, our sign-based thinking has been rapidly popularized and applied, so that the idea of EBN has been accepted and recognized by the majority of medical workers [29]. As a field of nursing, the development of EBN has gone through a long process, and it has been applied and popularized all over the country for a long time.

The concept of PDCA and EBN is integrated into the holistic nursing of the operating room [29, 30]. Regarding the traditional holistic nursing of the operating room, the application of the concept of PDCA and EBN in the ear, nose, and throat operating room can effectively prevent the incidence of hypothermia during operation and analyze the reasons: the occurrence of hypothermia suppresses the heat production center, and cold sensitive neurons excite muscle tremors to maintain body temperature balance and induce chills. Shivering increases discomfort and wound pain in patients. Patients with pain, pipeline stimulation, feeling discomfort, side effects of anesthetic drugs, lack of consciousness, anxiety and other factors are easy to cause restlessness [30]. Restlessness can cause patients to fall into bed, wound dehiscence, bleeding, and unplanned extubation. Meanwhile, the increase of heart rate and blood pressure caused by sympathetic nerve excitation can easily lead to cardio-cerebrovascular events, which seriously threaten the safety of operation [31]. The incidence of shivering and restlessness in this study group is significantly lower compared to the control group, which is similar to the conclusion of Sonia [32]. According to the traditional theory, postoperative patients need to have anal exhaust before they can eat. Long-term fasting can lead to intestinal mucosal atrophy, flora imbalance, nutrition lower than the needs of the body, affecting the rehabilitation of patients. Some scholars have also indicated that early eating does not cause nausea, vomiting, abdominal distension, diarrhea, and other discomfort and can shorten the first exhaust and defecation time [33]. In this study, based on the concept of PDCA and EBN, holistic nursing in the operating room was applied to patients in the ear, nose, and throat operating room. The clinical department developed a more detailed instruction manual for postoperative functional exercise (such as breathing exercise, effective cough, ankle pump exercise, straight leg elevation test, posture change “trilogy,” four-step turn-over, and six-part wake-up method), equipped with corresponding out-of-bed activity chairs to emphasize the participation of family members, which can reduce the sense of helplessness after operation, enhance the confidence of rehabilitation, help to enhance the compliance of postoperative rehabilitation exercise, promote the recovery of gastrointestinal function and venous reflux of lower extremities, and prevent postoperative pulmonary infection and venous thrombosis [34, 35].

In summary, it is effective to integrate the concept of PDCA and EBN into the holistic nursing of the operating room in the ear, nose, and throat operating room, which can effectively enhance the surgical indexes of the patients, reduce the incidence of postoperative infection, shorten the time of postoperative resuscitation and hospitalization, reduce the cost of hospitalization, and promote the satisfaction of surgical patients. While further multicenter studies are necessary, this series of nursing interventions remains worthy of replication in the clinical setting.

## Figures and Tables

**Figure 1:** Comparison of nursing satisfaction between two groups.

**Figure 2:** Comparison of the incidence of hypothermia, chills and restlessness between the two groups.

**Figure 3:** Comparison of the incidence of postoperative infection between the two groups.

**Table 1:** Comparison of related indexes in operating room between two groups of patients [$\bar{x}$ ± *s*].

Group	*N*	Extubation time of endotracheal tube (min)	PACU residence time (min)	Postoperative hospital stays (d)	Hospitalization expenses (yuan)	Operation time (min)
C group	100	48.49 ± 3.41	46.79 ± 4.31	5.29 ± 1.21	3653.91 ± 44.77	194.14 ± 3.55
R group	100	32.19 ± 4.42	37.48 ± 3.56	3.11 ± 1.35	2135.94 ± 34.22	143.85 ± 3.31
*t*		29.198	16.654	12.024	269.380	103.611
*P*		<0.01	<0.01	<0.01	<0.01	<0.01

**Table 2:** Comparison of nursing quality scores between the two groups [$\bar{x}$ ± *s*, points].

Group	*N*	Instrument and equipment management	Equipment preparation	Nurses' cooperation skills	Disinfection and isolation quality	Total score
C group	100	23.64 ± 2.32	15.12 ± 2.77	24.66 ± 2.56	15.12 ± 1.56	84.31 ± 1.66
R group	100	26.66 ± 2.23	18.55 ± 1.12	28.12 ± 1.66	19.55 ± 2.66	94.55 ± 2.31
*t*		9.384	11.479	11.340	14.365	35.998
*P*		＜0.01	＜0.01	＜0.01	＜0.01	＜0.01

**Table 3:** Comparison of individual quality control scores between two groups of clinical departments [$\bar{x}$ ± *s*, points].

Group	*N*	Ward management	Rescue and therapeutic articles	Drug management	Special nursing first-class nursing	Nursing documents
C group	100	85.53 ± 2.66	84.55 ± 1.31	85.93 ± 2.11	86.43 ± 1.55	86.54 ± 2.11
R group	100	92.12 ± 1.12	94.32 ± 1.53	91.85 ± 2.34	95.53 ± 1.35	94.42 ± 1.64
*t*		22.832	48.505	18.788	44.271	29.486
*P*		<0.01	<0.01	<0.01	<0.01	<0.01

## Data Availability

The datasets used and analyzed during the current study are unavailable due to the patient privacy.
